# Hematological Findings among COVID-19 Patients Attending King Khalid Hospital at Najran, Kingdom of Saudi Arabia

**DOI:** 10.1155/2022/4620037

**Published:** 2022-02-16

**Authors:** Ahmed M. E. Elkhalifa, Abozer Y. Elderdery, Ibrahim Ali Al Bataj, Abdelhakam G. Tamomh, Masaud M. Alyami, Hussein A. Almakrami, Mubarak A. Alofair, Mohammed A. Almorish, Salem Bashanfer, Mohammed I. Tabash, Hadeil M. E. Idris, Dania Z. Ahmed, Abdulaziz H. Alhamidi, Pooi Ling Mok

**Affiliations:** ^1^College of Health Sciences, Saudi Electronic University, Riyadh, Saudi Arabia; ^2^Faculty of Medical Laboratory Sciences, University of El Imam El Mahdi, Kosti, Sudan; ^3^College of Applied Medical Science, Jouf University, Sakaka, Saudi Arabia; ^4^Healthcare Model, General Directorate of Health Affairs-Najran, Saudi Arabia; ^5^Dhahran Aljnoob Health Sector-Asser, Saudi Arabia; ^6^Najran General Directorate of Health Affairs, Saudi Arabia; ^7^College of Medicine and Health Sciences, Sana'a University, Yemen; ^8^Centre for Regenerative Medicine, Institute for Regeneration and Repair, University of Edinburgh, Edinburgh, UK; ^9^Department of Laboratory Medicine, Faculty of Applied Medical Sciences, Al-Azhar University, Gaza, State of Palestine; ^10^College of Applied Medical Sciences, Shaqra University, Saudi Arabia; ^11^Hampshire Hospitals NHS Foundation Trust and Health Education, UK; ^12^Clinical Laboratory Sciences Department, College of Applied Medical Science, King Saud University, Riyadh, Saudi Arabia; ^13^Department of Biomedical Sciences, Faculty of Medicine and Health Sciences, Universiti Putra Malaysia, 43400 UPM Serdang, Selangor, Malaysia

## Abstract

COVID-19 is a global pandemic viral infection that has affected millions worldwide. Limited data is available on the effect of COVID-19 on hematological parameters in Saudi Arabia. This study is aimed at examining the role of hematological parameters among COVID-19 patients admitted to King Khalid Hospital in Najran, Saudi Arabia. This is a retrospective, hospital-based study of 514 cases who were recruited during August to October 2020. 257 COVID-19 patients formed the study group, and a further 257 negative subjects formed the control group. Anemia was significantly elevated in positive subjects over controls (respectively, 64.2% and 35.8%), with patients 2.5 times more likely to be anemic (*p* < 0.01). Thrombocytopenia was higher in patients over controls (respectively, 62% and 38%), with patients ~1.7 times more likely to be thrombocytopenic (*p* < 0.01). Moreover, leukopenia was significantly higher in patients over controls (respectively, 71% and 29%), with positive subjects ~2.6 times more likely to be leukopenic. Our study results indicate that mild anemia associated with leukopenia may have diagnostic value for COVID-19. Careful assessment of hematological parameters, at baseline and throughout the disease path, will assist physicians in formulating personalized approaches to treatment and promptly offer intensive care to those in greater need.

## 1. Background

Since the discovery of COVID-19, in Wuhan, China, on December 29th 2019, key questions have been raised on the potential of the relationship between its progression and various clinical and laboratory findings [1]. Dyspnoea, dry cough, weakness, fever, myalgia, and lymphopenia constitute the condition's most common symptom set, while pneumonia manifests in radiologic signs [2].

Secondary infections, respiratory distress, arrhythmia, acute heart damage, kidney failure, shock, and even death may present in severe cases [3–5]. Early diagnosis is vital immediately after admission, considering the high mortality rate and the short onset time of ARDS [4]. Hematological parameters associated with COVID-19 are variables drawn from various reports and are currently being utilized to predict outcome including mortality [6].

Full blood count (FBC) is inexpensive and not difficult to perform. Included in the FBC are various values, including counts of leucocytes (neutrophils and lymphocytes) and thrombocytes, indices of erythrocytes, and certain ratios of these values. Of leucocytes, the neutrophils are the most distinctive and essential component of the immune system. The role of lymphocytes in infections is well evidenced. Moreover, thrombocytes have a crucial role in the regulation of several inflammatory processes [4, 7, 8].

Interestingly, some studies report that COVID-19 infection is associated with haemoglobin (Hb) level reduction [9, 10], which is also seen in some pneumonias [11]. The leukocytes in blood circulation respond to stress by both increasing neutrophils and decreasing lymphocytes. Additionally, the ratio of these two values is used as an inflammation marker, as reported in a study by Huang and coworkers. They found a significant alteration in levels of two granular leucocytes (neutrophils and eosinophils) plus lymphocytes in COVID-19 patients, suggesting this as an indicator for disease presence, progression, and effectiveness of treatment [4]. For this reason, a study by Gothwal and coworkers recommended that the neutrophil-to-lymphocyte (NEU-LYM) ratio (NLR) could be used as a blood test as it might assist in the diagnosis of COVID-19 severity [12].

Furthermore, Liu et al. identified neutrophil-to-lymphocyte ratio as a risk factor for COVID-19 mortality in hospital patients. However, as admitted in the same paper, the usefulness of these markers/hematological parameters in terms of diagnosis has not been explored [13]. Although on a relatively small scale, Hu et al. recognised significant leukopenia in COVID-19 patients [14]. Limited data has been published on the hematological findings of COVID-19 positive patients in Saudi Arabia [15, 16]. This study has the objective of examining the characteristics of hematological parameters among positive patients compared with negative subjects at Najran City, King Khalid Hospital.

## 2. Methods

### 2.1. Research Design of Setting and Subject Set

A hospital-based, retrospective observational study was conducted at the King Khalid Hospital at Najran City, from August to October 2020, to compare hematological parameters of red blood cells (RBCs), platelets, and white blood cells (WBCs) among patients with and without COVID-19 diagnosis. In this study, 514 patients were recruited, a study group of 257 patients testing positive and a control group of 257 testing negative. Those who had blood and chronic diseases or who had taken drugs that could affect their complete blood picture were excluded from the control group. Infection was detected by a positive result of extracted nasopharyngeal swab samples analyzed using RT-PCR (Reverse Transcriptase Polymerase Chain Reaction) SARS-CoV-2 assay test at the clinical laboratory of King Khalid Hospital at Najran.

### 2.2. Data Collection

Ethical approval was obtained from the hospital administration and the local health authority. Clinical and demographic data plus hematological index values were excerpted from medical records of the clinical laboratory database. Hematological parameters were included, such as mean corpuscular volume, RBC and platelet counts, mean corpuscular Hb, and WBC count (total and differential). Following WHO criteria, anemia threshold was set at Hb < 11.5 g/dL, <12.0 g/dL, and <13.0 g/dL for children, nonpregnant females, and men, respectively [17]. Leukopenia was demarcated as total WBC count < 4.0 10^9^/L and thrombocytopenia as platelet count < 150.0 10^9^/L [18]. Demographic data included age, gender, and nationality, while the data included clinical signs and their severity.

### 2.3. Analysis of Data

IBM SPSS Statistics v26.0 was used to analyse the data. Qualitative variables were conveyed as proportions and frequencies. Tests of normality were done and normally distributed continuous data were presented as mean and standard deviation (SD). The mean values of the hematological indicators were evaluated using the independent sample *t*-test, and the association between COVID-19 positivity and hematological cytopaenias was tested using the Chi-square test. Statistical significance was demarcated at *p* values of ≤ 0.05.

### 2.4. Ethical Consideration

This research was granted approval by the Saudi Electronic University Institutional Ethics Committee, REC Number (SEUREC-CHS20113).

## 3. Results

### 3.1. Characteristics of the Study Patients

Table 1 shows that 171 (66.5%) of COVID-19 patients were male and 86 (33.5%) were female, while 156 (60.7%) of non-COVID-19 patients were male and 101 (39.3%) were female. The age range of COVID-19 patients was 20-90 years old; 153 of these (9.5%) between 30 and 60 years old, 81 (31.5%) over 60, and the remaining 23 (8.9%) below 30. The non-COVID-19 patients' age range was 20-88; 150 of these (58.4%) between 30 and 60, 48 (16.4%) over 60, and the remaining 45 (17.5%) below 30. 152 (59.1%) of the study group were Saudi citizens and the 105 (40.9%) from other nationalities, i.e., Yemeni, Egyptian, Sudanese, Bangladeshi, Pakistani, Filipino, Indian, and others. Regarding the clinical information of COVID-19 patients, 73 of them (28.4%) were attending the hospital in critical status, 56 (21.8%) with mild symptoms, 52 (20.2%) asymptomatic, 49 (19.1%) with moderate symptoms, and 27 (10.5%) with severe symptoms. Regarding the COVID-19 patients' situation during the study period, 182 (70.8%) recovered and were discharged from the hospital, 23 (8.9%) were still ICU patients at the end of the study period, 16 (6.2%) were isolated in hospital wards, and 36 (14%) unfortunately passed away. Furthermore, there was a highly significant correlation in status among COVID-19 patients with their age ($\underset{¯}{p}<0.001$), while the gender factor showed a nonsignificant association (*p* > 0.05) as explained in Table 2.

### 3.2. Hematological Indices Compared, between COVID-19 Positive and Negative Persons

The mean indices of Hb concentration (*p* < 0.001), MCH (*p* < 0.001), MCHC (*p* < 0.001), and MCV (*p* = 0.004) were all significantly lower in COVID-19 positive patients compared with negative, while the RDW was significantly higher (*p* = 0.002). In contrast, the RBC count showed only a nonsignificant difference (*p* = 0.113).

The mean indices were significantly lower for counts of lymphocytes (*p* < 0.001), monocytes (*p* < 0.001), and thrombocytes (*p* < 0.001) among cases testing positive, while the neutrophil count was significantly elevated (*p* < 0.001). The TWBC count (*p* = 0.609) and the mean platelet volume (*p* = 0.296) showed only a nonsignificant difference (*p* = 0.113), as shown in Table 3.

### 3.3. Hematological Cytopaenias Compared, between COVID-19 Positive and Negative Persons

The prevalence of anemia was significantly elevated in patients with COVID-19 compared with those without (controls), respectively, at 64.2% and 35.8%. On the one hand, cases were 2.5 times more likely to be anemic; on the other, the prevalence of thrombocytopenia was significantly elevated in cases over controls, respectively, at 62% and 38%, where cases were 2.6 times more likely to be leukopaenic, as explained in Table 4.

## 4. Discussion

The prevalence of COVID-19 cases has seen an increase globally. Assessing clinical, demographic, and hematological indicators is important when investigating the COVID-19 outbreak. Few studies have investigated hematological parameters associated with COVID-19 within Saudi Arabia. Thus, our study investigated hematological parameters such as RBCs, platelets, and WBCs among cases with and without COVID-19. This included a total of 514 patients from King Khalid Hospital, Najran City, Saudi Arabia, of which 257 were COVID-19 patients.

Our study provides extensive details on demographic data and hematological parameters in hospitalized patients during an outbreak in Najran. Of all the 257 patients with COVID-19 diagnosed, 171 (66.5%) were males, and 86 (33.5%) were females, this resembling previous data where males and females were 69.3% and 30.7%, respectively [19]. While another recent review (meta-analysis) of 3,111,714 documented global cases found that there was no difference among both males and females with confirmed COVID-19 [20], which is similar to our finding association (*p* value = 0.112). Similarly to previous studies, more males had COVID-19 than females (66.5% and 33.5%, respectively) [16, 21]. However, gender showed no significant association (*p* value = 0.112). This may be attributed to the effect of immunological differences between genders or behavioural choices [16]. Moreover, previous studies have also indicated that males are more susceptible to COVID-19 than females and have accounted for this in terms of the lower expression in females of angiotensin-converting enzyme-2 receptors for coronavirus. Lifestyle is also a factor, including that in males' levels of both smoking and drinking are increasing; also, women have culturally more accountable mindsets regarding the pandemic. Interestingly, there are the immunological variations based on sex and regulated by sex hormones and X chromosomes [22]. COVID-19 seems to kill more men than women as in this study; 29 males (17.0%) have died compared to 7 females (8.1%); this is also similar to the two most hard-hit Caucasians; as found that in Italy, most of the COVID-19 deaths occurred in males, while in Spain, almost twice as many men died as women [16, 23]. Other studies also reported that Chinese data first showed a gender disparity in deaths, where 41.9% of admitted patients were women and the majority of deaths being of men [24, 25]. The average age of COVID-19 patients was 52.85 ± 15.89, indicating that COVID-19 targeted individuals in their 60s, and those in that age group are at greater risk of serious illness than individuals in their 20s-50s. Our current study shows that age is significantly associated with COVID-19 (*p* value = 0.001). In contrast, the mean age of positive cases was slightly older than the mean age reported within other studies conducted in Saudi Arabia [16, 26]. This is also contradicted by a previous study which suggested that this condition affects a younger age range inside Saudi Arabia [20]. The mortality rate of older patients was significant and very high at 27.2% compared to the other groups 13.0% and 7.2%. In another meta-analysis, 6,111,583 subjects were reviewed. 141,745 (23.2%) were aged 80 years or older. In patients under 50 years, average mortality was <1.1%, the highest being in the UK (20.8%) and the lowest in China (3.2%), whereas in New York it increased exponentially with age (20.9%) [27]. Yanez et al. have also reported that patients aged 65 or older had a substantially higher COVID-19 mortality rate in the 16 countries studied. However, younger males had a higher risk of COVID-19 death over younger females, where 77% of fatalities were men [28]. COVID-19 cases were found to have significantly lower levels of Hb concentration MCH, MCHC, and MCV in comparison with negative patients, this result being quite similar to that of previously reported studies [20, 29]. This could be associated with the action of the virus against the development or degradation of RBC or the existence of comorbidities. Moreover, a study by Thomas and coworkers reported that COVID-19 RBCs showed decreased levels of main antioxidant (PRDX1, SOD1, G6PD) enzymes and increased markers of degradation of proteins [30]. COVID-19 patients revealed significantly elevated levels of RDW compared to patients testing negative. In a previous study, higher levels of RDW were identified in patients with severe compared to moderate symptoms [31]. Similarly, to previous research, RBC count had no significant indication in COVID-19 patients [32]. The present study also showed that there was no significant difference in total RBCs and mean platelet volume, while neutrophil, lymphocyte, monocyte, and platelet counts were significant. By contrast, in a study by Guan and coworkers, 1,099 cases documented that the percentage of lymphocyte was low in ~83% of cases at admission [24]. Lymphocytopenia was also detected more frequently in severe cases than nonsevere, at 96.1%. Additionally, low numbers of thrombocytes were present in 36.2% of all patients, with severe cases showing it more frequently at 57.7%. These results concur with findings from a number of previous studies showing that the infection severity could be associated with low lymphocytes and thrombocytes [4, 5, 33, 34]. The mean indices of lymphocyte count, monocyte count, and platelet count were significantly lower in positive than negative patients (*p* < 0.001 for all). Upon hematological analysis, a low lymphocyte count in positive patients has been commonly noted in previous studies [29, 32]. Furthermore, leucopaenia prevalence was elevated significantly, by a factor of 2.6. Although lymphopenia may be quite common among COVID-19 patients, leucopaenia has also previously been reported [35]. Platelets and lymphocytes are an important part of inflammatory responses, with previous studies highlighting the association of a low platelet count and lymphocytes in the disease severity of COVID-19 [32, 35]. Theoretical postulations consider a low platelet count as an indicator for thrombocytopenia; however, further research is needed. Noteworthily, reports also indicate that COVID-19 patients can show varying WBC counts [35]. Alongside a low platelet count, previous studies identified thrombocytopenia as an indicator of disease severity in COVID-19 cases [35, 36]. Thrombocytopenia prevalence was significantly elevated compared with non-COVID-19 patients (62% vs. 38%, respectively), where the former were approximately 1.7 times more likely to be thrombocytopenic. Moreover, COVID-19 patients showed a significantly higher neutrophil count than the non-COVID-19 group (*p* value < 0.001). This was consistent with previous research as indicated that an increased neutrophil count is correlated with disease severity in positive COVID-19 [26, 32].

## 5. Conclusion

To conclude, this study highlighted and compared hematological parameters of RBCs, platelets, and WBCs of COVID-19 cases. This saw reduced levels of lymphocytes, platelets, and increased neutrophil count in positive patients compared to negative. It thereby recognises the importance of these parmeters in diagnosis of the disease. Identifying abnormal hematological parameters and continuous observation can also be essential in the disease progression of COVID-19.

## Figures and Tables

**Table 1:** Characteristics of studied patients.

Characteristics	COVID-19 patients (*N* = 257)	Non-COVID-19 patients (*N* = 257)
	*N* (%)	*N* (%)
Gender		
Male	171 (66.5)	156 (60.7)
Female	86 (33.5)	101 (39.3)
Age (years)		
<30	23 (8.9)	45 (17.5)
30-60	153 (59.5)	150 (58.4)
>60	81 (31.5)	62 (24.1)
Mean SD	52.85 15.89	48 16.4
Range	20-90	20-88
Nationality		
Saudi	152 (59.1)	152 (59.1)
Yemeni	28 (10.9)	21 (8.2)
Egyptian	12 (4.7)	7 (2.7)
Bangladeshi	23 (8.9)	15 (5.8)
Pakistani and Filipina	15 (5.8)	22 (8.6)
Indian	8 (3.1)	8 (2.7)
Others	19 (7.4)	33 (12.8)
Symptoms		
Asymptomatic	52 (20.2)	NA
Mild	56 (21.8)	NA
Moderate	49 (19.1)	NA
Severe	27 (10.5)	NA
Critical	73 (28.4)	NA
Current situation		
Recovered	182 (70.8)	NA
Isolated at hospital wards	16 (6.2)	NA
ICU patient	23 (8.9)	NA
Passed away	36 (14)	NA

**Table 2:** Current situation among COVID-19 patients and related factors in the King Khalid Hospital at Najran City, Saudi Arabia (2020).

Characteristics	Current situation (*N* = 257)				*χ* ^2^	*p* value
	Recovered	Isolated	ICU	Pass away		
	*N* (%)	*N* (%)	*N* (%)	*N* (%)		
Gender						
Male	114 (66.7)	13 (7.6)	15 (8.8)	29 (17.0)	5.99	.112
Female	68 (79.1)	3 (3.5)	8 (9.3)	7 (8.1)		
Age (years)						
<30	16 (69.6)	2 (8.7)	2 (8.7)	3 (13.0)	23.87	0.001
30-60	123 (80.4)	9 (5.9)	10 (6.5)	11 (7.2)		
>60	43 (53.1)	5 (6.2)	11 (13.6)	22 (27.2)		

**Table 3:** Hematological indices among COVID-19 patients and non-COVID-19 patients attending the King Khalid Hospital at Najran City, Saudi Arabia (2020).

Indices	COVID-19 patients (*N* = 257)	Non-COVID-19 patients (*N* = 257)	*t*	*p* value
	M (±SD)	M (±SD)		
Hb (g/dL)	12.5 (1.76)	12.96 (1.5)	3.19	0.001
RBC (10^12^/L)	4.76 (0.72)	4.67 (0.6)	1.58	0.113
MCV (fL)	83.98 (9.7)	86.1 (6.9)	2.86	0.004
MCH (pg)	26.55 (3.5)	27.98 (2.7)	5.17	<0.001
MCHC (g/dL)	31.53 (2.7)	32.47 (1.4)	5.01	<0.001
RDW (%)	15.7 2.96	15.06 (2.2)	3.13	0.002
WBC count (10^9^/L)	8.22 (5.59)	8.44 (3.6)	0.511	0.609
Neutrophil (%)	69.09 (17.4)	58.81 (17.0)	6.94	<0.001
Lymphocyte (%)	22.4 (14.0)	29.28 (13.5)	5.62	<0.001
Monocyte (%)	7.1 (3.4)	8.6 (3.2)	5.23	<0.001
Platelet (10^9^/L)	262.1 (112.4)	309.7 (128.2)	4.47	<0.001
MPV (fL)	9.3 (1.40)	9.1 (1.23)	1.04	0.296

**Table 4:** Hematological cytopaenias among COVID-19 patients and non-COVID-19 patients in the King Khalid Hospital at Najran City, Saudi Arabia (2020).

Hematological abnormality	COVID-19 patients (*N* = 257)	Non-COVID-19 patients (*N* = 257)	OR (95% CI)	*p* value
	*n* (%)	*n* (%)		
Anemia	120 (64.2)	67 (35.8)	2.5 (1.71-3.59)	<0.001
Thrombocytopenia	31 (62.0)	19 (38.0)	1.7 (0.94–3.12)	0.074
Leukocytopenia	32 (71.0)	13 (28.9)	2.6 (1.36–5.21)	0.003

## Data Availability

The data used to support the findings of this study are included within the article.
